The article "Modified Activated Carbon: A Supporting Material for Improving Clostridium beijerinckii TISTR1461 Immobilized Fermentation" was retracted in 2024. Reasons: signs of a paper mill; suspected computer-generated content; unreliable results or conclusions; concerns about the data.

# Modified Activated Carbon: A Supporting Material for Improving *Clostridium beijerinckii* TISTR1461 Immobilized Fermentation

**DOI:** 10.1155/2023/3600404

**Published:** 2023-03-23

**Authors:** Piyawat Chinwatpaiboon, Akarin Boonsombuti, Thanyalak Chaisuwan, Ancharida Savarajara, Apanee Luengnaruemitchai

**Affiliations:** ^1^The Petroleum and Petrochemical College, Chulalongkorn University, Bangkok 10330, Thailand; ^2^Department of Materials Science, Faculty of Science, Srinakharinwirot University, Bangkok 10110, Thailand; ^3^Department of Microbiology, Faculty of Science, Chulalongkorn University, Bangkok 10330, Thailand; ^4^Center of Excellence on Catalysis for Bioenergy and Renewable Chemicals (CBRC), Chulalongkorn University, Bangkok 10330, Thailand

## Abstract

This study aimed to investigate the effect of activated carbon (AC) as an immobilization material in acetone-butanol-ethanol fermentation. The AC surface was modified with different physical (orbital shaking and refluxing) and chemical (nitric acid, sodium hydroxide and, (3-aminopropyl)triethoxysilane (APTES)) treatments to enhance the biobutanol production by *Clostridium beijerinckii* TISTR1461. The effect of surface modification on AC was evaluated using Fourier-transform infrared spectroscopy, field emission scanning electron microscopy, surface area analyses, and X-ray photoelectron spectroscopy, while the fermented broth was examined by high-performance liquid chromatography. The chemical functionalization significantly modified the physicochemical properties of the different treated ACs and further enhanced the butanol production. The AC treated with APTES under refluxing provided the best fermentation results at 10.93 g/L of butanol, 0.23 g/g of yield, and 0.15 g/L/h of productivity, which were 1.8-, 1.5-, and 3.0-fold higher, respectively, than that in the free-cell fermentation. The obtained dried cell biomass also revealed that the treatment improved the AC surface for cell immobilization. This study demonstrated and emphasized the importance of surface properties to cell immobilization.

## 1. Introduction

Fossil fuels, the main sources of transportation energy in Thailand over the last century, are being gradually replaced by more environmentally friendly and sustainable biofuels [1, 2]. Thailand is pledged to reduce greenhouse gas emissions in the energy and transportation sectors by 156.86 MtCO_2_eq by 2030. Among the most rational candidates for alternative energy sources in Thailand, biofuel is one of the sustainable energies that can be adopted to meet the energy needs of the automobile industry. Typically, bioethanol is blended with gasoline at various ratio compositions at retail pumps: gasohol 95, gasohol 91, E10, and E20 [3]. Recently, biobutanol has gained a lot of interest, being a better fuel than bioethanol due to its higher energy density, air-fuel ratio, octane number, lower heat of vaporization, less corrosiveness, less hygroscopic, and lower vapour pressure, and it can also be blended with gasoline at any ratio [1, 4, 5].

Butanol (butyl alcohol or C_4_H_9_OH) is a hydrocarbon containing four-carbon atoms with an alcohol functional group [4, 6]. Typically, biobutanol is produced by acetone-butanol-ethanol (ABE) fermentation using *Clostridium* spp. (e.g., *C. acetobutylicum*, *C. beijerinckii*, *C. pasteurianum*, *C. sporogenes*, *C. saccharoperbutylacetonicum*, and *C. saccharobutylicum*) with an ABE production mass ratio of 3 : 6 : 1 [1, 4, 6]. The ABE fermentation is an anaerobic process having two major phases: acidogenesis and solventogenesis. During the acidogenesis phase, *Clostridium* sp. converts carbon sources to organic acids (acetic and butyric acids), and these are then consumed to produce solvents (acetone, butanol, and ethanol) in the solventogenesis phase [1, 4]. In free cell cultures, *Clostridium* sp. is significantly affected by environmental stresses, such as the pH, temperature, solvents, salts, inhibitors, poisons, and self-destruction. [7]. Previous studies have indicated that the growth of *Clostridium* sp. will be suppressed when the butanol concentration is greater than 7.4 g/L [1, 2, 8, 9], and this low obtained butanol concentration will increase the cost of downstream purification. The complicated metabolism of ABE fermentation and inappropriate environment is the cause of cell membrane rupture [1, 10] and results in the low butanol concentration, yield, and productivity.

In order to alleviate these limitations, it was found that immobilization of the bacteria cells on a suitable supporting material could improve the microbial tolerance, yield, and ABE productivity [6, 11, 12]. The immobilized culture has a high cell density and can be applied to batch, fed-batch, and continuous fermentations [6, 7, 11]. For instance, ABE fermentation using *C. beijerinckii* immobilized on alkaline-treated Napier grass produced a high butanol concentration (8.99 g/L), which was 25% higher than that in a free cell culture [13]. The potential supporting material for cell immobilization should be inexpensive, stable, reusable, and nontoxic [7]. Many inorganic and organic materials have been used as supports, such as celite [14], sand [14], brick [14], glass beads [15], clay [16], ceramics [17], plastics [18], alginate [19], zeolite [20], lignocellulosic material [13], and activated carbon (AC) [21, 22]. The porous nature of AC with its high surface area and high adsorption capacity makes it a promising material for bacterial immobilization [22]. However, previous studies reported that an immobilized *Clostridium* sp. culture on AC produced a lower butanol concentration compared to the free-cell system [23], although the reason for this was unclear.

Modifications of the physicochemical properties of the support surface play an important role to cell immobilization. There are various methods for surface modification or functionalization, such as treatment with acid, alkaline, silylation, ammonia, and ozone [24–27]. In this study, the AC was treated with three chemical treatments: nitric acid (HNO_3_), sodium hydroxide (NaOH), and (3-aminopropyl) triethoxysilane (APTES) via two physical methods (orbital shaking and refluxing) to modify the morphology and surface functional groups (such as carboxyl, carbonyl, phenol, quinone, and lactone groups) [24, 25]. The acid treatment will increase the acidic and hydrophilic properties of the AC surface, while the alkaline treatment will enhance its basic property [26]. Silylation is one of the treatments that introduces basic groups, such as -NH_2_, with physical attractions and/or covalent bonds between the AC surface and APTES-NH_2_ groups [27]. The use of APTES modification has also been reported for bacterial immobilization on cellulase [28] and protein [29].

In this study, the treatment of AC as a carrier for the immobilization of *Clostridium beijerinckii* TISTR1461 was evaluated in terms of the butanol yield and compared to that obtained in a free cell batch fermentation. During the ABE fermentation, the broth was collected to monitor the changes in the medium and products using high-performance liquid chromatography (HPLC). At the end of fermentation, the broth and immobilized supporting materials were collected and dried to find the respective cell biomass in each fermentation system. These treatments could improve the surface and overall properties of the AC, resulting in increased cell adsorption and butanol production capacities. The physicochemical properties of the untreated and various treated AC samples were characterized by field emission scanning electron microscopy (FE-SEM) equipped with energy-dispersive X-ray (EDX), Brunauer–Emmett–Teller (BET) surface area (*S*_BET_) analysis, Fourier-transform infrared spectroscopy (FT-IR), and X-ray photoelectron spectroscopy (XPS) analyses.

## 2. Materials and Methods

### 2.1. Carrier Treatments

Raw AC with a 4–12 mesh particle size was supplied from DARCO® (Sigma-Aldrich Co., Ltd.). Before treatment, the AC was washed with deionized water, dried, and sieved to a 12-mesh particle size (1.68 mm). The raw AC was then treated at a 1 : 10 (w/v) AC: liquid ratio with different physical (orbital shaking and refluxing) and chemical (HNO_3_, NaOH, and APTES) treatments. The physical treatment was performed by two different apparatuses: orbital shaking and refluxing methods.

For the chemical treatments, concentrated HNO_3_ (65%, QReC) was used as the acid solution [30], while 1 M NaOH, prepared by dissolving 40.40 g NaOH pellets (99%, MERCK) in 1000 mL of deionized water [30], was used as the alkali solution. For the APTES solution, about 2.65 mL APTES (99%, Sigma Aldrich) was mixed with 100 mL ethanol (99.9%, QReC).

The AC was treated by soaking in HNO_3_ with orbital shaking at 60°C for 6 h [30]. After that, the untreated and acid-treated samples were reacted with NaOH for 6 h [30] and denoted as SH_S_ and NASH_S_, respectively. For the refluxing method, the AC was refluxed in APTES or NaOH at 78°C for 6 h [31, 32] and denoted as APTES_R_ and SH_R_, respectively. Then, the SH_S_, NASH_S_, and SH_R_ samples were washed with deionized water until the washings were at a neutral pH. For the APTES_R_, the sample was washed several times with ethanol [32]. The samples were then dried in the oven at 105°C overnight and kept in a desiccator prior to further analysis or use as an immobilized material.

### 2.2. Preparation of the *C. beijerinckii* Inoculum

The *C. beijerinckii* TISTR1461 culture was activated in a cooked meat medium (Difco™ laboratories, USA) supplemented with 20 g/L glucose (10 mL) in a 25 mL screw-capped bottle and then incubated at 37°C in an anaerobic jar for 48 h [13, 20, 32]. The resultant culture was transferred to P2 medium (60 g/L glucose, 1 g/L yeast extract, 0.5 g/L KH_2_PO_4_, 0.5 g/L K_2_HPO_4_, 2.2 g/L CH_3_COONH_4_, 1 mg/L para-amino-benzoic acid, 1 mg/L thiamin, 0.01 mg/L biotin, 0.2 g/L MgSO_4_•7H_2_O, 10 mg/L MnSO_4_•H_2_O, 10 mg/L FeSO_4_•7H_2_O, and 10 mg/L NaCl, pH 6.5) [33, 34] (93 mL) in a 250 mL screw-capped bottle and incubated at 37°C in an anaerobic jar for 48 h [13, 20].

### 2.3. ABE Fermentation

The *C. beijerinckii* TISTR1461 inoculum was inoculated into a P2 medium (100 mL in 250 mL screw-capped bottle) to an initial optical density at 600 nm (OD_600 nm_) of 0.3 (1.03 g/L dried cell biomass) [13]. For the immobilized cultures, the untreated or treated AC was sterilized by autoclaving at 121°C for 15 min and then added at 2% (w/v) into the P2 medium inoculum. The culture was then purged with 99.99% nitrogen gas (N_2_) at a 10 mL/min flow rate for 5 min [13] and incubated at 37°C, 150 rpm orbital shaking for 120 h. The pH was not controlled in this study throughout the fermentation process. At 0, 12, 24, 48, 72, 96, and 120 h of incubation, the sample was collected, centrifuged (25°C for 20 min at 8000 rpm with RCF up to 14490 × g), filtered through a 0.22 *µ*m membrane, and kept at −20°C [13]. Resultant supernatant was analyzed for the concentrations of residual glucose, organic acids, and butanol.

After 120 h of incubation, the cell biomass from the broth and the respective (untreated or treated) AC carrier was collected and dried until at a constant weight. These cell biomasses were recorded as the suspended and immobilized dry weight, respectively, and reported as the dry weight of cells (*g*) divided by the volume of fermentation broth (*L*) [35].

### 2.4. Characterization

In order to examine the pH of AC, the samples were shaken with 2% (w/v) of 0.1 M sodium nitrate (NaNO_3_) solution [30]. After 48 h, the pH was measured with a glass pH electrode and a pH meter (Eutech instrument; model: pH700).

The physicochemical properties of AC were examined by FE-SEM using a Hitachi S-4800 microscope equipped with energy-dispersive X-ray (EDX) analysis for elemental identification. The sample was dried and sputter-coated with platinum to minimize the electrostatic charge, and then located on a sample holder using a carbon tape. The morphological images were obtained by applying a 15 kV accelerating voltage [13].

To observe the surface colonization, the SEM proceeded with a JEOL JSM-5410LV microscope operated at an acceleration voltage of 15 kV. The immobilized materials were collected at the end of fermentation and fixed in 2.5% (w/v) glutaraldehyde (in 0.1 M phosphate buffer and pH 7.4) for 2 h. Next, the samples were cleaned by 0.1 M phosphate buffer in order to remove all the precipitated cells and washed with water. The samples were then dehydrated in a graded ethanol series (30%, 50%, 70%, 95%, and 100% (v/v)) and dried in a critical point dryer. Finally, the samples were fixed to stubs using conductive silver paint and sputter-coated with a thin layer of gold [13, 20].

The *S*_BET_ of the samples was analyzed by N_2_ adsorption/desorption measurements using an Autosorb-1 Gas Sorption surface area analyzer (Quantachrome Corporation) using the BET method. A sample of 0.5 g was degassed under a vacuum atmosphere at 110°C for 24 h to eliminate any moisture and contaminant adsorbed on the sample surface [30].

The FT-IR spectra of each sample were measured on a Thermo Nicolet, NEXUS 670 instrument (ThermoScientific, USA) over the range of 4000-400 cm^−1^ at a spectral resolution of 4 cm^−1^ and using 64 scans. Prior to the analysis, the sample was ground with dried potassium bromide (KBr) at a (w/w) ratio of 1 : 100 and pressed into pellets at 10 tons for 5 min.

The XPS surface analysis was employed to determine the oxidation states of C1s, N1s, and O1s using a Kratos Axis Ultra DLD photoelectron spectrometer equipped with a magnetic immersion lens and charge neutralizer. Monochromatic Al K*α* was used as the X-ray source at 15 kV. The residual pressure in the ion-pumped analysis chamber was lower than 5 × 10^7^ torr. The binding energy was referenced to the C1s peak (284.6 eV) to account for the effects of charging [36, 37].

### 2.5. Analytic Procedures

The bacterial growth and cell biomass were determined by optical density at 600 nm (OD_600 nm_) using a UV-VIS Spectrometer (UV-1800; Shimadzu, Japan). Sterilized water was used as the blank and dilutant.

The residual glucose and organic acids from the resultant supernatant were analyzed using HPLC (Shimadzu, Japan), equipped with an Aminex-HPX 87H column (300 mm × 7.8 mm, Bio-Rad Lab, USA), deashing cartridge holder (30 mm × 4.6 mm, Bio-Rad Lab, USA), and microguard cation H+ refill cartridge holder (30 mm × 4.6 mm, Bio-Rad Lab, USA). The HPLC conditions were a 60°C column temperature, 5 mM sulphuric acid (H_2_SO_4_) as the mobile phase at 0.6 mL/min, and detected by a refractive index detector (RID-20A; Shimadzu, Japan) at 40°C [13, 20]. The injection volume was 50 *μ*L.

The butanol yield and dried cell biomass were calculated according to equations (1) and (2), while the butanol enhancement over that obtained in the free cell culture was obtained from equation (3):

(1) $$\begin{array}{c} Butanol\;yield\;=\;\frac{Butanol}{Consumed\;glucose}\left[g/g\right], \end{array}$$

(2) $$\begin{array}{c} Dried\;cell\;biomass\;=\;\frac{Dried\;weight\;of\;cell}{Fermentation\;broth}\left[g/L\right], \end{array}$$

(3) $$\begin{array}{c} Enhanced\;butanol\;=\;\frac{Butanol_{system}-\;Butanol_{Freecell}}{Butanol_{Freecell}}\;x\;100\;\left[\%\right]. \end{array}$$

## 3. Results and Discussion

### 3.1. Materials Characterization

The AC was treated by different physical (orbital shaking and refluxing methods) and chemical (HNO_3_, NaOH, and APTES) methods before using as an immobilized material. The treatments played an important role on the physicochemical properties of the carrier, which then affected the butanol production obtained from the ABE fermentation.

Representative FE-SEM images of the morphology of various AC samples are shown in Figure 1. The different physical treatment methods affected the surface morphology of the treated AC samples. Micrographs in Figures 1(a)–1(c)) reveal the details of morphology in which the surface features of the treated AC samples were significantly different from those of the untreated AC. Figures 1(b)–1(e)) show that the particle size of AC treated with NaOH by a refluxing method was smaller than when treated by orbital shaking. The refluxing method results in more severe conditions, due to the applied direct shear force (magnetic agitation) and higher temperature, which results in the destruction of the AC's matrix. After treatment, the external surface was much more accessible due to the corrosion of scattered fragments and creation of some cleavages and cracks.

The N_2_ adsorption-desorption isotherms, pore size distribution, and S_BET_ of all the samples are exhibited in Figures S1 and S2 and Table 1, respectively. The presence of mesopores was evidenced by the hysteresis loop of capillary condensation, which appeared from *p*/*p*_0_ = 0.45 to 1. A pore size distribution between 3 and 5 nm was clearly seen. The morphology results corresponded to the *S*_BET_ results (Table 1), in which the *S*_BET_ of samples changed after treatment. The BET results showed that the two-steps (HNO_3_ and NaOH) treated sample (NASH_*S*_) had the highest surface area (574 m^2^/g), a 17% increase over the untreated AC. However, the *S*_BET_ of the SH_*S*_ sample was lower than the untreated AC sample. The previous studies have reported that alkaline treatment reduced the surface area and micropore volume because the pores were enlarged after treatment [24, 25, 37]. This agreed with the reduction in the pore volume of SH_S_ and SH_R_ in this study, as shown in Table 1. The APTES_R_ showed the lowest surface area of 306 m^2^/g because the large molecule of APTES might block some pores [32], resulting in a reduced effective surface area and pore volume. The X-ray diffraction (XRD) patterns of the untreated and different treated AC samples (Figure S3) revealed no significant changes in the AC samples after different treatments.

The pH of immobilized materials is also one of the factors that strongly influences microorganisms [1, 38]. The carbon pH of the AC is related to the existence of acidic and basic functional groups on its surface. Table 1 shows the carbon pH of the untreated and different treated AC, suggesting that the different chemical treatments were moderately successful. According to Brönsted acids' behaviour, Park and Jang mentioned that the chemical treatments developed the hydroxyl groups to be protonated, neutral, and ionized surface hydroxyl groups (AC-OH_2_^+^, AC-OH, and AC-O^−^, respectively) [25]. The results showed that the carbon pH of the different treated AC samples was higher than that of the untreated AC (Table 1) because the acidic characters were decreased after chemical treatment. The HNO_3_ treatment produced some acidic groups, such as carboxyl acid and quinine groups, on the surface [26], which corresponded to the experimental result of the primary treatment of AC with HNO_3_ (NA_S_) that had as carbon pH of 3.78 (not shown in Table 1).

However, the dominant acidic groups on the surface can form an inappropriate environment for microorganisms leading to their death, including for *C. beijerinckii* TISTR1461 as it has an optimum condition of around pH 6-7 at 37°C [1, 13, 20]. To decrease the acidity, the NaOH treatment was performed so that Na^+^ replaced the H^+^ of the surface acid groups [26]. As a result, the carbon pH of the alkaline-treated samples (SH_S_, NASH_S_, and SH_R_) was evidently higher than the untreated AC. The treatment with APTES also reduced the acidic character resulting in the highest carbon pH (pH 8.47). Comparing between different operating methods, the NaOH treatment with refluxing had a slightly higher carbon pH than that with orbital shaking (pH 7.19 and 6.65, respectively). This implied that refluxing had a superior efficiency to react the acidic groups on the carbon surface than orbital shaking.

The molecular components and structures were evaluated by FT-IR analysis. The surface functional groups of AC were changed by the chemical treatments (Figure 2). The peak was around 780 cm^−1^ related to C-H bending and C-H stretching vibration [39]. The untreated AC exhibited the carboxylic acid groups as the small bands at 1700 and 3300 cm^−1^ from the carboxyl groups to hydroxyl groups, respectively, [24, 30, 40]. After the treatment with NaOH, the acidic surface groups were neutralized [40], resulting in a reduced 1700 cm^−1^ band and an increase of 3300 cm^−1^ band. The appearance of a small peak after the NaOH treatment at around 1410 cm^−1^ suggested a lactone structure [24, 40]. These results agreed well with a previous study of NaOH-treated AC prepared from olive stones, which showed an enhanced basic nature (mostly in the phenolic categories) [41], the formation of lactone in phenolic groups by alkaline treatment [30].

From Figure 2(c), the two-stage treated AC (NASH_S_) had peaks near 1600 and 1700 cm^−1^ indicating quinone and carboxyl structures, respectively [40]. The appearance of these peaks implied that some acids in the micropores were not neutralized by the NaOH treatment [24, 40]. Acid treatment increased the level of acidic surface groups, while the alkaline treatment reduced the level of carboxyl surface groups [40]. Positively charged acid groups (H^+^) were produced by the HNO_3_ treatment, and then the NaOH treatment replaced the H^+^ of acid groups by Na^+^, resulting in a reduced acidity [26, 40]. The spectra of APTES_R_ revealed that not only was O-H bonding formed on the surface but also the N-H stretching vibration occurred, resulting in an increment in the 3300 cm^−1^ band intensity [39, 42]. A small peak around 2920 cm^−1^ was assigned to C-H stretching vibration [31, 42], and the small peak around 1550–1610 cm^−1^ was associated with N-H and C=N vibration [26, 39, 42]. Some studies suggest that the peak around 1200–1260 cm^−1^ is due to Si-CH_2_ stretching [42] and Si-O-Si [43]. The change in the functional groups on the surface of treated-AC samples agreed with the measured carbon pH (Table 1).

For APTES treatment, the APTES molecule was hydrolysed into alkylammonium, hydroxide, and carboxylate ions (equation (4)) [44, 45]. These ions might interact and graft on the AC's surface, as shown schematically in Figure 3(b) [27], in accordance with the FT-IR results. The chemical composition of the sample's surface was examined by XPS analysis on the differences in their binding energies. To clarify the APTES treatment, the chemical states of the untreated and APTES-treated AC were analyzed and compared by XPS, with the fitting curves of C1s, N1s, and O1s signals shown in Figure 4.

(4) $$\begin{array}{c} \begin{array}{c} {{\text{H}}_{2}\text{N}-\left({\text{CH}}_{2}\right)}_{3}-Si-{\left(C_{2}H_{5}O\right)}_{3}\\ APTES \end{array}\;+\;\begin{array}{c} 3{\text{H}}_{2}\text{O}\\ Water \end{array}\;\overset{hydrolysis}{\to }\;\begin{array}{c} {{\text{H}}_{2}\text{N}-\left({\text{CH}}_{2}\right)}_{3}-Si-{\left(OH\right)}_{3}\\ Alkylammoniumion \end{array}\;+\;\begin{array}{c} 3{\text{C}}_{2}{\text{H}}_{5}\text{O H}\\ Ethanol \end{array} \end{array}$$

The XPS spectra revealed substantial changes in the nature of the untreated and APTES_R_ samples (Figure 4(a)). The different bonding states of carbon correspond to the aromatic and aliphatic C-C/C-H (284.5 eV), C-O (285.8 eV), and O-C=O (289.5 eV) [27, 42, 43, 46]. For the untreated AC, the peak of carbon linked to oxygen at 289.5 eV was ascribed to carboxyl groups [26]. The XPS spectra of N1s showed no significant peaks, indicating that there were no nitrogen bonds before treatment. The fitting of the O1s spectrum showed a single peak at 532.4 eV, which was ascribed to ether-like C-O-C groups [42, 43, 46]. After the APTES treatment (Figure 4(b)), the C1s signals displayed broad peaks at 284.6 eV for aromatic and aliphatic C-C/C-H [27, 42, 46], 285.6 eV for C-O, C-N [42], and 288.5 eV for carbon linked to oxygen (O-C-O, O-C=O) [42] and aliphatic carbon linked to nitrogen (N-CO-N) [43, 46]. The N1s spectra displayed two signals at 398.2 eV (free amino and C-N-H) [42, 43] and 400.3 eV (protonated amine and C-N^+^) [42]. Compared to the untreated sample, the APTES_R_ sample showed a higher O1s intensity referring not only to C=O [42, 43] but also to Si-O-H [44, 47]. The contribution of the peak at 532 eV of the treated sample was significantly increased, compared to AC, probably due to the successful anchoring of the carbon-APTES surface. These results indicate the formation of chemical bonds between APTES and the surface of the AC.

In addition, the atomic composition of various samples, as evaluated by EDX analysis, is shown in Table 2. Compared to the untreated AC, the carbon composition of the treated samples decreased slightly (around 10%) while the oxygen composition increased 1.6- to 2.0-fold which is in an agreement with the FT-IR and XPS analyses.

### 3.2. ABE Fermentation by *C. beijerinckii* TISTR1461 in a Free Cell Culture

Over the first 12 h of the free cell culture, *C. beijerinckii* TISTR1461 utilized glucose for rapid growth (Figure 5(a)) with the production of organic acids, as shown by the rapid decrease in the culture pH from 6.30 to 5.35 (Figure 5(b)). Thus, *C. beijerinckii* TISTR1461 was in the acidogenic phase, in accordance with previous reports [1, 4]. From 12 to 48 h of incubation, the concentration of organic acids decreased obviously, whereas the concentration of solvents increased (Figures 5(b) and 5(c)). This indicated that *C. beijerinckii* TISTR1461 shifted from the acidogenic to the solventogenic phase, where glucose, acetic acid, and butyric acid were utilized to produce solvents (acetone, butanol, and ethanol) with butanol as the major product [4]. From 48 h of incubation onwards, there was a slight decrease in the level of glucose, organic acids, solvents, and culture pH. The maximum level of total solvents produced was 8.13 g/L, comprised of acetone 1.89 g/L, butanol 6.10 g/L, and ethanol 0.14 g/L.

### 3.3. ABE Fermentation by *C. beijerinckii* TISTR1461 Immobilized on Various Types of Treated AC

After 120 h of incubation, the immobilized *C. beijerinckii* TISTR1461 on the untreated AC exhibited a slightly higher cell biomass (1.36 g/L; Table 3) but lower butanol level (2.98 g/L; Figure 6), while the free cell culture yielded a cell biomass of 1.13 g/L (Table 3) and butanol level of 6.10 g/L (Figure 5). The higher cell biomass of immobilized untreated-AC culture than in the free cell culture might due to porous structure of the untreated AC providing a higher surface area for cells to adsorb [22]. However, only 43% of the glucose was utilized by the immobilized culture on the untreated AC compared to 62% by the free cell culture. The low level of glucose consumption and the low butanol production indicated that the untreated AC did not provide an appropriate environment for *C. beijerinckii* TISTR1461 to grow and produce butanol. Some previous studies mentioned that immobilization of *Clostridium* sp. on AC might change the bacterial metabolism to produce by-products (CO_2_ and H_2_) rather than butanol [35, 48].

For the fermentation with various treated AC samples, the results are exhibited in Figure 6. The immobilized culture of *C. beijerinckii* TISTR1461 on the different treated ACs showed a lower residual glucose level but higher cell biomass and butanol formation than in the free cell and untreated AC culture. The cell biomass and butanol production of the cultures immobilized on the different treated ACs were ranked (from high to low) as APTES_R_ > SH_R_ > NASH_S_ > SH_S_ (Table 3). The ACs treated under orbital shaking (SH_S_ and NASH_S_) produced organic acids at levels (2.11 and 2.41 g/L, respectively) as high as those in the free cell culture (2.24 g/L), whereas in the ACs treated under refluxing (SH_R_ and APTES_R_), the organic acid levels were 1.5- and 1.8-fold higher than in the free cell culture, respectively. The production of both organic acids and butanol from the treated ACs under refluxing was higher than in those treated under orbital shaking.

With respect to the production of organic acids and butanol, SH_R_ produced a higher level of organic acids (3.46 g/L) and butanol (7.61 g/L) than SH_S_ because SH_R_ had a higher surface area and lower acidity (higher carbon pH). For the immobilized fermentation with APTES_R_, a 1.8-fold higher butanol concentration (10.93 g/L) was produced than in the free cell culture. The microorganisms might create an amide bond and develop a biofilm on the surface of the APTES_R_ [11, 12]. The biofilm then protects the *C. beijerinckii* TISTR1461 from environmental stresses and so results in an increased cell tolerance and butanol production. Previous studies about immobilized cellulase [28] and protein [29] on APTES surface also showed similar trends. In addition, in this study, an increased dried cell biomass was found on all the immobilized AC systems compared to in the free cell fermentation (Table 3), which was due to the chemical bond or electrostatic force between the microorganisms and the treated-AC's surface.

In the ACs treated under orbital shaking (SH_S_ and NASH_S_), *C. beijerinckii* TISTR1461 cells grew as suspended cells at the same level as immobilized cells, while in the reflux-treated AC cultures (SH_R_ and APTES_R_), the proportions of immobilized cells were 8.3- and 9.7-fold higher than the suspended cells, respectively (Table 3). This indicated that chemical or electrostatic bonds between cells immobilized on SH_R_ and APTES_R_ might be stronger than those on SH_S_ and NASH_S_. The highest cell biomass was noted on APTES_R_ (three-fold higher than in the free cell culture), and so APTES_R_ likely provided the most favourable environment for *C. beijerinckii* TISTR1461.

The results obtained from the present study using *C. beijerinckii* TISTR1461 immobilized on the different treated ACs in this study are compared with those obtained with other immobilized materials from other studies in Table 4. The observed butanol concentrations were in the range of 1.42–10.93 g/L, and the highest butanol concentration was obtained in this work using the APTES_R_ with an initial glucose concentration of 60 g/L. The highest butanol productivity of 0.20 g/L·h was observed with immobilized *C. acetobutylicum* on PHBwet jet. However, it is very difficult to compare and find an ideal material to achieve both a high butanol concentration and productivity.

The SEM images (Figure 7) confirmed the immobilization of *C. beijerinckii* TISTR1461 on/into the various types of treated ACs. The dimension of *Clostridium* sp. cells has previously been reported to be about 500 nm diameter and 2-3 *μ*m length [35], so the bacteria can move and grow through the cracks of the treated AC samples (Figure S4).  Figure S5 displays the extracellular component (white thin thread) between the bacteria (rod-shaped) and the treated AC surface, indicating a successful cell immobilization on the carrier.

## 4. Conclusion

Surface modification of AC before using it as a carrier for *C. beijerinckii* TISTR1461 can be critical for its ability to promote cell adhesion and ABE fermentation. The characterization of the treated ACs confirmed the improvement of their physical and chemical properties, exhibiting changes in the *S*_BET_ and functional groups on the carbon surface. Among the different treatments, the AC treated by APTES under refluxing (APTES_R_) exhibited the lowest surface area, but the immobilized fermentation with this carrier produced the highest butanol concentration (10.93 g/L) at some 1.8-folds more than in the free cell culture. Thus, the chemical properties of the carrier's surface are likely to play a more important role in cell immobilization than the physical properties. Overall, AC with a high surface area and protonated amine grafting on the surface could be an attractive material for immobilizing *Clostridium* cells in culture. Further studies using this technique in continuous fermentation to improve the productivity and production of biobutanol are warranted.

## Figures and Tables

**Figure 1:** Representative FE-SEM images at 1000x magnification of the (a) untreated (AC), (b) SH_S_, (c) NASH_S_, (d) SH_R_, and (e) APTES_R_ samples. Images shown are representative of those seen from at least three such fields of view and three independent samples.

**Figure 2:** Representative FT-IR spectra of the (a) untreated AC, (b) SH_S_, (c) NASH_S_, (d) SH_R_, and (e) APTES_R_ (condition: range of 400–4000 cm^−1^ with 8 cm^−1^ resolution).

**Figure 3:** Schematic representation of APTES modification of AC: (a) APTES molecule and (b) APTES on the AC's surface.

**Figure 4:** Representative peak-fitting XPS of the (1) C1s, (2) N1s, and (3) O1s signals of the (a) untreated AC and (b) APTES_R_ (Condition: performed under a high vacuum condition (≤5 × 10^7^ torr), calibrated by reference to the C1s peak at 284.6 eV).

**Figure 5:** The ABE fermentation by *C. beijerinckii* TISTR1461 free cell culture showing the levels of the (a) cell biomass and residual glucose, (b) pH, acetic, butyric, and total acids, and (c) acetone, butanol, and ethanol. Data are shown as the mean ± SD, derived from three replicated independent samples.

**Figure 6:** The ABE fermentation by *C. beijerincki*i TISTR1461 immobilized on various treated ACs (untreated SH_S_, NASH_S_, SH_R_, and APTES_R_) showing the levels of (a) residual glucose, (b) pH, (c) total acids, and (d) butanol. Data are shown as the mean ± SD, derived from three replicated independent samples.

**Figure 7:** Representative SEM images (7500x magnification) of (a) SH_S_, (b) NASH_S_, (c) SH_R_, and (d) APTES_R_ after 120 h of batch fermentation showing the colonization of *C. beijerinckii*. Images shown are representative of those seen from at least three such fields of view and three independent samples.

**Table 1:** Physical properties of the untreated and treated activated carbons.

Sample	Carbon pH	Surface area (m^2^/g)	Pore volume (mL/g)	Pore size (nm)
**Untreated**	5.20	491	0.59	3.81
**SH**_**S**_	6.65	470	0.54	3.88
**NASH**_**S**_	5.96	574	0.66	3.89
**SH**_**R**_	7.19	517	0.57	3.91
**APTES**_**R**_	8.47	306	0.40	3.87

**Table 2:** The EDX derived atomic percentage of the untreated and treated ACs.

Sample	C	O	S	Others
**Untreated**	88.24	6.24	1.08	4.44
**SH**_**S**_	78.54	10.18	1.35	9.93
**NASH**_**S**_	78.99	12.25	0.00	8.76
**SH**_**R**_	79.86	12.07	1.10	6.97
**APTES**_**R**_	78.27	11.96	1.66	8.11

**Table 3:** Dried cell biomass of *C. beijerinckii* TISTR1461 in ABE fermentation when cultivated as free cells and immobilized cell cultures on the untreated and treated AC samples.

Cultivation	Dried cell biomass (g/L)					
	Start (0 h)			End (120 h)		
	Suspended	Immobilized	Total	Suspended	Immobilized	Total
Free cell	1.03 ± 0.11	0.00 ± 0.00	1.03 ± 0.11	1.13 ± 0.07	0.00 ± 0.00	1.13 ± 0.07
Immobilized cell						
Untreated	1.03 ± 0.11	0.00 ± 0.00	1.03 ± 0.11	0.93 ± 0.12	0.43 ± 0.09	1.36 ± 0.21
SH_S_	1.03 ± 0.11	0.00 ± 0.00	1.03 ± 0.11	1.00 ± 0.01	1.20 ± 0.09	2.20 ± 0.09
NASH_S_	1.03 ± 0.11	0.00 ± 0.00	1.03 ± 0.11	1.10 ± 0.30	1.30 ± 0.08	2.40 ± 0.38
SH_R_	1.03 ± 0.11	0.00 ± 0.00	1.03 ± 0.11	0.31 ± 0.07	2.60 ± 0.47	2.91 ± 0.54
APTES_R_	1.03 ± 0.11	0.00 ± 0.00	1.03 ± 0.11	0.34 ± 0.05	3.30 ± 0.33	3.64 ± 0.38

Data are shown as the mean ± SD, derived from three replicated independent samples.

**Table 4:** Comparison of ABE fermentation (batch-fermentation) from *Clostridium spp.* immobilized on various carriers.

Carrier	Strain	Medium	Butanol				Ref.
			Concentration (g/L)	Yield (g/g)	% Enhanced from free cell	Productivity (g/L/h)	
DARCO® AC:	*C. beijerinckii* TISTR1461	P2 medium (glucose 60 g/L)	(Free cell fermentation produced 6.10 g/L of butanol)				This work
Untreated			2.98	0.11	−50.15	0.04	
SH_S_			6.42	0.15	+5.42	0.09	
NASH_S_			7.05	0.16	+15.57	0.10	
SH_R_			7.61	0.17	+24.75	0.11	
APTES_R_			10.93	0.23	+79.18	0.15	
Brick	*C. beijerinckii* TISTR1461	P2 medium (glucose 60 g/L)	5.80	0.16	+9.64	0.12	[20]
Zeolite 13X			8.58	0.16	+62.19	0.12	
AC	*C. acetobutylicum* ATCC 824	(Glucose 27–35 g/L)	3.83	0.11	−32.22	0.09	[23]
Sugarcane bagasse			5.80	0.24	+2.47	0.16	
Brick			4.92	0.20	−13.07	0.15	
AC	*C. acetobutylicum* CICC 8012	P2 medium (glucose 30 g/L)	3.38	0.11	−40.23	0.07	[35]
Bagasse			5.80	0.24	+2.47	0.18	
Brick			4.92	0.20	−13.07	0.15	
Poly(3-hydroxy-butyrate) (PHB)	*C. acetobutylicum* ATCC 824	RCM-s medium (glucose 60 g/L)					[49]
PHB solvent casting			5.40	∼0.25	−41.30	0.11	
PHB wet jet			9.70	0.28	+5.43	0.20	
PHB electrospining			9.10	∼0.20	−1.08	0.19	
Brick	*C. acetobutylicum* BCRC 10639	(Glucose 60 g/L)	∼10.53	—	−6.48	0.15	[50]
Sponge			∼1.42	—	−87.39	0.02	
Nonwoven fabric			∼9.95	—	−11.63	0.14	

## Data Availability

The data used to support the findings of this study are included in the article. Further data or information required are available from the corresponding author upon reasonable request.

## Supplementary Materials

Supplementary Materials Supplementary Figures S1, S2, and S3 provide the N_2_ adsorption-desorption isotherms, BJH pore size distribution, and XRD patterns of the untreated and treated AC samples, respectively. The SEM images of all the treated AC samples are shown in Figures S4. *C. beijerinckii* TISTR1461 cells immobilized on the treated AC samples are shown in Figures S5.
